# A Unified Model Using Distantly Supervised Data and Cross-Domain Data in NER

**DOI:** 10.1155/2022/1987829

**Published:** 2022-05-29

**Authors:** Yun Hu, Hao He, Zhengfei Chen, Qingmeng Zhu, Changwen Zheng

**Affiliations:** ^1^Institute of Software, Chinese Academy of Sciences, Haidian, Beijing 100190, China; ^2^University of Chinese Academy of Sciences, Haidian, Beijing 100190, China; ^3^Shenzhen Power Supply Bureau Co., Ltd., Shenzhen 518001, China

## Abstract

Named entity recognition (NER) systems are often realized by supervised methods that require large hand-annotated data. When the hand-annotated data is limited, distantly supervised (DS) data and cross-domain (CD) data are usually used separately to improve the performance. The distantly supervised data can provide in-domain dictionary information, and the hand-annotated cross-domain information can be provided by cross-domain data. These two types of information are complemental. However, there are two problems required to be solved before using directly. First, the distantly supervised data may contain a lot of noise. Second, directly using cross-domain data may degrade performance due to the distribution mismatching problem. In this paper, we propose a unified model named PARE (PArtial learning and REinforcement learning). The PARE model can simultaneously use distantly supervised data and cross-domain data as external data. The model uses the partial learning method with a new label strategy to better handle the noise in distantly supervised data. The reinforcement learning method is used to alleviate the distribution mismatching problem in cross-domain data. Experiments in three datasets show that our model outperforms other baseline models. Besides, our model can be used in the situation where no hand-annotated in-domain data is provided.

## 1. Introduction

Name entity recognition [1] as a fundamental natural language processing (NLP) task has received significant attention. The NER system tries to label each word in sentences with predefined types, such as brand and product. The results of NER can be used in many downstream NLP tasks, such as coreference resolution [2], relation extraction [3], and question answering [4]. The supervised methods are often used to realize the NER system [5–7]. However, supervised methods often require large annotated data. In practice, obtaining hand-annotated data can be a very expensive and laborious process. When limited hand-annotated data is accessible, distantly supervised data and cross-domain data are widely used as external resources [8–11].

The distantly supervised data is obtained by the matching method. An example is shown in Figure 1. The word “Samsung” is matched by the entity dictionary. More in-domain data can be obtained through distant supervision. Cross-domain data can provide compensative information. The cross-domain learning methods utilize the high resource domain information to improve the low resource domain performance [10]. It is natural to combine these two types of data.

However, there are some problems with directly using two types of data. First, in distantly supervised data, when a word is not matched by the entity dictionary, the word has no clear label. The matching method can lead to many errors. In Figure 1 (we use Chinese as a case of study; however, in order to better make readers understand, Chinese characters are not allowed in the figure, and we translate Chinese to English), the label of the word “mobile” should be product. Previous work uses a word-level method and a sentence-level method to alleviate errors [8]. In the word-level method, the partial learning method is used. In the sentence-level method, the reinforcement learning method is used. In the traditional partial learning method, the labels of the words are the whole label set when the words are not contained in the entity dictionary. For example, the label of “mobile” has 5 candidate labels (\{“B-Brand,” “I-Brand,” “B-Product,” “I-Product,” “O”\}). However, the traditional label strategy does not consider label features in NER. For example, the label of “mobile” cannot be “I-Brand.” Second, in cross-domain learning, the parameter sharing method is a widely used method [10, 12]. However, directly using the parameter sharing method may lead to performance reduction due to the distribution mismatching [13]. Previous works mainly focus on using different network architectures to capture private features and shared features [14]. In addition, these works cannot handle the situation where no hand-annotated domain data is provided.

In this paper, we explore a PARE model which can simultaneously use distantly supervised data and cross-domain data as external data. For distantly supervised data, we use a new label strategy considering label features of NER. The new label strategy can reduce redundant labels in the partial learning method. In cross-domain data, the reinforcement learning method is used to alleviate the distribution mismatching problem in the parameter sharing method. We evaluate our PARE model in three datasets and show that our methods outperform other baseline models. Besides, our PARE model can be used in the situation where no hand-annotated in-domain data is provided. We only use distantly data and cross-domain data as inputs and achieve competitive results. Contributions of our work can be summarized as follows:

- We propose a PARE model. The PARE model can use distantly supervised annotated data and cross-domain data as external data simultaneously in Chinese NER.
- We propose an improved partial learning method to process distantly supervised NER data, which can better process the noise in distantly supervised data.
- We use the reinforcement learning method to process cross-domain NER data, which can alleviate the distribution mismatching problem in the parameter sharing method.

## 2. PARE Model

The architecture of the PARE model is shown in Figure 2. The model can be divided into three parts: core NER part, DS data selector part, and CD data selector part. The improved partial learning method is used in the core NER part to reduce the noise in distant supervision. The DS data selector part and CD data selector part are similar to those in [8, 13]. The DS data selector removes the noise sentence by reinforcement learning. The CD data selector selects the relevant sentence in the cross-domain dataset, which reduces the domain distribution mismatching. Through reinforcement learning, we can use the distantly supervised data and cross-domain data as external data simultaneously.

### 2.1. Core NER

The core NER is based on the LSTM-CRF model [7], which is widely used in named entity recognition. The core NER part contains three subparts: embedding layer, Bi-LSTM layer, and CRF layer. The input of the model is a sentence *x*={*x*_1_, *x*_2_,…, *x*_*n*_}. *x*_*i*_ is the word in sentence and *x* can be from hand-annotated data, distantly supervised data, or cross-domain data. The output of the model is *y*={*y*_1_, *y*_2_,…, *y*_*n*_}, which is the label of sentence *x*. To better process the distantly supervised data, a new label strategy is proposed in core NER.

#### 2.1.1. Embedding Layer

We use the embedding layer as the first step of a neural network model. The embedding layer maps the word into a low dimensional dense vector, which contains the semantics of the word. The embedding vector *e*_*i*_ can be obtained as

(1) $$\begin{array}{c} e_{i}=\text{Embedding}\left(x_{i};\theta_{e}\right), \end{array}$$

where *x*_*i*_ is the input word and *θ*_*e*_ is the embedding table. The embedding layer can also use an additional contextualized word embedding such as BERT [15]. *e*_*i*_ is concatenated with the output of BERT.

#### 2.1.2. Feature Extractor

The feature extractor uses the output of word embedding. We use the Bi-LSTM as the feature extractor. The LSTM can handle gradient vanishing/exploding problems well as shown in previous work [16]. A common LSTM unit is composed of a cell, an input gate, an output gate, and a forget gate. The Bi-LSTM concatenates forward LSTM output and backward LSTM output to capture information from context [17]. The output of Bi-LSTM *h*_*i*_ can be represented as

(2) $$\begin{array}{c} h_{i}=\text{Bi}-\text{LSTM}\left(e_{i};\theta_{l}\right), \end{array}$$

where *θ*_*l*_ is the parameters in Bi-LSTM.

#### 2.1.3. CRF

We use Conditional Random Fields (CRF) to predict the label sequence, because the neighborhood information can be considered in CRF. For example, CRF considers that the “I-Product” cannot be behind the “B-Brand.” For a sentence *x* and one possible label sequence *y*, we define the score to be

(3) $$\begin{array}{c} \text{score}\left(x,y\right)=\overset{n}{\underset{i=0}{\sum }}A_{y_{i},y_{i+1}}+\overset{n}{\underset{i=1}{\sum }}P_{i,y_{i}}, \end{array}$$

where *A* is a matrix of transition score. *A*_*i*,*j*_ represents the score of a transition from the tag *i* to tag *j*. *P* is the matrix of the output score. *P* matrix can be obtained by using a feed-forward neural network after the Bi-LSTM output. The probability of the sequence *y* can be obtained by

(4) $$\begin{array}{c} p\left(y|x\right)=\frac{e^{\text{score}\left(x,y\right)}}{\sum_{\bar{y}\in A\left(y\right)}e^{\text{score}\left(x,\bar{y}\right)}}, \end{array}$$

where *A*(*y*) is all candidate label sequences.

The traditional CRF can process hand-annotated data and cross-domain data well because every word in hand-annotated data and cross-domain data has an explicit label. For distantly annotated data, if the words are in the dictionary, the words have explicit labels. In traditional label strategy, if the words are not in the entity dictionary, the labels are the whole label set. For example, the word “mobile” will have 5 labels. The partial learning method can better process these label strategies. For the input sentence *x*, there will be a set of possible label sequence *C*(*y*), because every word will have several labels. We compute the probability of the all possible predicted sequence *C*(*y*) by summing the probability of each possible label sequence $\hat{y}$:

(5) $$\begin{array}{c} p\left(C\left(y\right)|x\right)=\frac{\sum_{\hat{y}\in C\left(y\right)}e^{\text{score}\left(x,\hat{y}\right)}}{\sum_{\bar{y}\in A\left(y\right)}e^{\text{score}\left(x,\hat{y}\right)}}. \end{array}$$

However, the previous label strategy does not consider label features in NER. Consider that the whole label set may lead to many redundant labels. The redundant labels may harm the model performance. In this paper, we use a new label strategy. The new label strategy removes some impossible labels. Some label features are shown as follows:

- The start label cannot be “I-XXX.” “XXX” represents an entity type, like “Brand.” For example, the label of “I” cannot be “I-Brand” or “I-Product” in Figure 1.
- The label of punctuation is “O.”
- The label “I-YYY” cannot be after the label “B-XXX” or “I-XXX.” “YYY” represents another entity type. For example, the label of “mobile” cannot be “I-Product” in Figure 1.

By using the new label strategy, the number of possible label sequences (*|C*(*y*)*|*) may reduce, and the performance may increase. During training, the log probability of the correct sequence log(*p*(*C*(*y*)*|x*)) is maximized. During decoding, the output sequence is given by

(6) $$\begin{array}{c} y^{*}=\underset{y\in A\left(y\right)}{\text{arg}\max}\text{score}\left(x,y\right). \end{array}$$

### 2.2. Data Selector

The data selector uses reinforcement learning method to select proper sentences. The overall training procedure is shown in Algorithm 1. In each epoch, we first select the cross-domain data and then select the distantly supervised data. Before doing the selection process, the hand-annotated data is merged with distantly supervised data and cross-domain data to obtain the merged data, respectively. To obtain more feedback, we divide the merged data into many random-size bags. Every sentence in bags obtains a state. During the selection process, for each sentence from distantly supervised data, the DS data selector has an action to decide whether to select the sentence or not. The CD data selector has an action to decide whether to select the cross-domain sentences or not. We directly select the sentences from the hand-annotated dataset. After doing the selection process in a bag, different selections will lead to different rewards. The DS reward is used as the feedback of the DS data selector and updates the DS data selector. The CD data selector is also updated through the domain reward. The goal of data selectors is to maximize the reward when the data selectors take action. After doing the whole selection process in dataset, the selected sentences are used to train the core NER, which can obtain the new state and reward in reinforcement learning. After the training processing, the core NER can be used as the NER system, which combines the distantly supervised data and cross-domain data information.

Some details of the reinforcement learning method are shown as follows. We use superscript *t* to discriminate different data and different data selectors. *t* can be {ds, *do*}, where ds, *do* mean distantly supervised and cross-domain, respectively.

#### 2.2.1. State

The state *s*^*t*^ can be the input of the selector network. For different data inputs, the model has the same pattern to obtain the state. The state *s*^*t*^ of the sentence contains the following information: (a) the serialized feature representation, which is extracted by the Bi-LSTM; (b) the label score is equal to *P* in equation (3).

#### 2.2.2. Policy Network

For each state *s*^*t*^, the action space *a*^*t*^ is \{0, 1\}. “1” represents selecting the sentence, and “0” represents not selecting the sentence. For DS annotated data, the action *a*_*i*_^ds^ is obtained from the DS data selector. The action *a*_*i*_^*do*^ is obtained from the CD data selector in cross-domain data. The data selector *π*_*θ*_^*t*^(*s*_*i*_^*t*^, *a*_*i*_^*t*^) is a multilayer perceptron with the parameter *θ*^*t*^. A logistic function is used as the policy function:

(7) $$\begin{array}{c} \pi_{\theta }^{t}\left(s_{i}^{t},a_{i}^{t}\right)=a_{i}\sigma \left(W^{t}*s_{i}^{t}+b^{t}\right)+\left(1-a_{i}^{t}\right)\left(1-\sigma \left(W^{t}*s_{i}^{t}+b^{t}\right)\right), \end{array}$$

where *W*^*t*^ and *b*^*t*^ are the parameters of selector. *σ*() is the sigmoid function.

#### 2.2.3. Reward

The reward is used to evaluate the quality of the selection. The reinforcement learning method in cross-domain has a different reward compared with reinforcement learning method in distant supervision because the goal of the selection is different. The goal of the DS data selector is to select the sentences which have less noise. The goal of the CD data selector is to select sentences that are relevant to hand-annotated data.

For distantly supervised data, when all the selections in the current merged data bag are finished, a delayed average reward is obtained. The selected distantly supervised sentences and hand-annotated sentences are used to compute the reward:

(8) $$\begin{array}{c} r^{\text{ds}}=\frac{1}{\left|{\hat{X}}^{\text{ds}}\right|+\left|X^{\text{ha}}\right|}\left(\sum \log\;p\left(C\left(y\right)|{\hat{x}}^{\text{ds}}\right)+\sum \text{log }p\left(y|x^{\text{ha}}\right)\right), \end{array}$$

where ${\hat{x}}^{\text{ds}}$ is the selected sentences, $\left|{\hat{X}}^{\text{ds}}\right|$ is the number of the selected sentences, *x*^ha^ is the hand-annotated sentences, and |*X*^ha^| is the number of the selected sentences. $\text{log }p\left(C\left(y\right)\;|\;{\hat{x}}^{\text{ds}}\right)$ and log *p*(*y* *|* *x*^ha^) are computed by equation (5).

The goal of the CD data selector is to select relevant sentences that fit the distribution of the target domain. For cross-domain data, we also obtained a delayed average reward. A reward is the distance between the selected domain data and hand-annotated data. We describe a simple distance in this paper, and the complex and better distance will be discussed in the future. The reward is set as

(9) $$\begin{array}{c} r^{do}=-d\left(\Phi \left({\hat{X}}^{do}\right),\Phi \left(X^{\text{ha}}\right)\right). \end{array}$$

The negative sign means that the distance value is small when the selected sentences are similar to the hand-annotated sentences. We use the maximum mean discrepancy to measure the distance. $\Phi \left({\hat{X}}^{do}\right)$ is the elementwise average of selected cross-domain sentences' state ${\hat{s}}^{do}$. Φ(*X*^ha^) is the elementwise average of hand-annotated sentences' state *s*^ha^.

Selector training: the policy gradient method [18] is used to optimize the policy network. The agents obtain the reward when all the actions have been done. For each bag, the feedback of every action *r*^*t*^(*a*_*i*_^*t*^) is equal to the average reward *r*^*t*^. The selector is updated as follows:

(10) $$\begin{array}{c} \theta^{t}=\theta^{t}+\alpha \overset{\left|{\hat{X}}^{t}\right|}{\underset{i=1}{\sum }}r^{t}\left(a_{i}^{t}\right){▽}_{\theta }\text{log}\pi_{\theta }^{t}\left(s_{i}^{t},a_{i}^{t}\right), \end{array}$$

where $\left|{\hat{X}}^{t}\right|$ is the number of selected sentences from distantly supervised data or cross-domain data.

### 2.3. No Hand-Annotated In-Domain Data

Our model can be used in the situation where only distantly supervised data and cross-domain data are provided. The motivation is that we can use cross-domain data instead of in-domain hand-annotated data. The details are shown in Algorithm 2. First, we use the distantly supervised data to select cross-domain data because the cross-domain data selection does not require the hand-annotated in-domain data to obtain the reward. Then, we use the selected cross-domain data to select the distantly supervised data. Finally, we use the selected cross-domain data and selected distantly supervised data to train the core NER part.

## 3. Experiments and Results

### 3.1. Datasets

Three hand-annotated in-domain datasets are used to evaluate our methods: e-commerce (EC) dataset, news dataset, and broadcast conversation (BC) dataset. The number of sentences is shown in Table 1. The EC dataset and news dataset are from [8] (the only difference is that we consider three types of entities (Brand, Product, and Model) in the EC dataset because cross-domain EC data has these common label types). The cross-domain data of the EC dataset is the Taobao dataset in [19]. For news data, the cross-domain data is the Chinese web text domain data from OntoNotes [20]. We also use a new dataset to evaluate our methods. For BC data, we randomly select 3000 sentences as train data, 500 sentences as development data, and 1000 sentences as test data from the OntoNotes Chinese broadcast conversation dataset [20]. The distantly supervised data is obtained from the rest of the OntoNotes Chinese broadcast conversation dataset. The construction method is similar to that in [8]. The cross-domain data is from OntoNotes Chines web data [20]. 6000 cross-domain sentences are used.

### 3.2. Parameters Setting

The pretrained embedding is shown to be helpful in previous works [7]. In core NER, the embedding is pretrained using word2vec [21] in a large user-generated text corpus. The embedding dimension is 100. The dimension of the LSTM is set to 100. The optimization method is RMSprop [22]. The initial learning rate is 0.001. The dropout rate is 0.2. The minibatch is 128. The max-epoch iteration is 500. For DS data selector and CD data selector, the dimension of the hidden layer in the multilayer perceptron is 100. The optimization method is Adam [23]. The initial learning rate is 0.001.

### 3.3. Results

For evaluation, the entity-level metrics of Precision (P), Recall (R), and their F1 score are used in this paper.

#### 3.3.1. Baseline

Eight baselines are considered to compare with our proposed model:

- LSTM-CRF (Hand) [7]: the model only uses the hand-annotated in-domain data as input.
- DS-PA-RL (Hand + DS) [8]: the model uses distantly supervised data as external data. The traditional partial learning method is used to process the distantly supervised data. The reinforcement learning method is used to delete the noise sentences. The code is the same as in [8].
- CD-SHA (Hand + CD) [24]: the model uses cross-domain data as external data. We mix cross-domain data with hand-annotation in-domain data as input data and then share all model parameters to train the model.
- CD-ADV (Hand + CD) [14]: the model uses cross-domain data as external data. An adversarial network is used to process the private and shared information between target domain and source domain.
- BERT-CRF (Hand) [15]: the model uses the hand-annotated in-domain data as input. The BERT is used as a context embedding encoder, and CRF is used as a decoder.
- SoftLexicon (Hand) [25]: the model uses the hand-annotated in-domain data as input and can capture the lexicon information through a segmentation label set.
- SCDL (Hand + DS) [26]: the distantly supervised data is used as external data, and a self-collaborative denoising learning method is used to handle label noise in distantly supervised data.
- Multicell (Hand + CD) [27]: the cross-domain data is used as external data, and different label types are processed by different cells in Multicell LSTM.

Four systems can be built based on our method:

- DS-IPA-RL (Hand + DS): the model uses the distantly supervised data as external data. Compared with [8], the model uses the new label strategies in the partial learning method.
- CD-RL (Hand + CD): the model uses cross-domain data as external data. The reinforcement learning method is used to select the relevant sentences in high resource domain.
- PARE (Hand + DS + CD): the PARE model uses distantly supervised data and cross-domain data simultaneously.
- PARE-BERT (Hand + DS + CD): the PARE-BERT uses the output of BERT as contextualized word embedding. Distantly supervised data and cross-domain data are used simultaneously.

The results of the models are shown in Table 2. We first analyze the models using traditional word embedding. From Table 2, the models using external data yield improvement compared with the LSTM-CRF model using hand-annotated data as input. This shows that using external data can be very helpful when hand-annotated data is limited. Different ways of using external resources will lead to different effects. The DS-IPA-RL model outperforms the DS-PA-RL model, showing that the new label strategies are helpful in the partial learning method. The CD-ADV model obtains worse results than the CD-SHA model. The reason may be that the CD-ADV model cannot utilize the CRF information sharing when the output label of the source domain and target domain are the same. The CD-RL model achieves the best performance compared with other cross-domain models. The PARE model achieves the best performance of all models. This indicates that our PARE model can utilize different external data well.

The Pretrained Language Model (PLM) has achieved competitive performance in the NER task, and our model is orthogonal with PLM. The results of models using BERT embedding are shown in Table 2. We can observe that our model can also improve the performance in the BERT situation. The results also show that PARE-BERT outperforms other baseline models using BERT. However, the improvement rate is smaller compared with the models without BERT. The reason may be that the language model has contained much information and the information gain brought by the unified model is relatively small.

To better analyze the different parts of the model, we divide our PARE model into some small parts to evaluate our methods. First, we will analyze the effect of using the label strategy in the partial learning method. Then, we evaluate the reinforcement learning method in cross-domain learning methods. Finally, we show the results in the situation where no hand-annotated data is provided.

#### 3.3.2. Improved Partial Learning

We compare the new label strategy with two label strategies and do not consider the influence of reinforcement learning. The first is the FA label strategy. In the FA label strategy, for the word that is not contained in the entity dictionary, the label is “O.” To utilize the FA data, we use the simple LSTM-CRF model [7]. The second is the PA label strategy. For the word that is not contained in the entity dictionary, the label is the whole label sets. We use the LSTM-CRF-PA model to utilize the PA data [8]. The results are shown in Table 3. The results show that the models using external data do not always obtain better results than the model only using hand-annotated data. Different label strategies achieve various results. The model using the IPA label strategy obtains the best results compared with the other models using hand-annotated and distantly supervised data. These facts show that label strategy is very important when distantly supervised data is used, and our new label strategy can be more effective than other label strategies.

#### 3.3.3. Cross-Domain Learning

In Table 4, we explore the performance of the model compared with the CD-SHA model. The CD-SHA model uses different amounts of randomly selected domain data. From the table, the CD-RL model outperforms the CD-SHA model using all domain data. This indicates that the reinforcement learning method can select relevant sentences and reduce negative transfer. The table can also show that the CD-RL model achieves the best results compared with the CD-SHA model using different amounts of domain data. These facts show that reinforcement learning selection is better than random selection.

#### 3.3.4. No Hand-Annotated In-Domain Data

Our PARE model can be extended to no hand-annotated situation. The model only uses distantly supervised data and cross-domain data as input, which greatly reduces the time of manual annotation. The training method is shown in Section 2.3. We compare our methods with three baselines:

- *LSTM-IPA*. The model uses only distantly supervised data as input. The improved label strategy is used to process the distantly supervised data.
- *SHA*. The model uses cross-domain data as input to train the model, and we directly transfer the model from the source domain to the target domain.
- *SHA-IPA*. The model uses distantly supervised data and domain data as input. The model is the same as that in [8], and we use domain data instead of hand-annotated in-domain data.

The results in three different datasets are shown in Table 5. From the table, we find that directly using distantly supervised data achieves very low performance. The reason can be that the data only from the distantly supervised method contains a lot of noise, especially the low coverage. The results of the SHA model are slightly better than those of the LSTM-IPA model. The SHA-IPA achieves the best results among all models. These facts show that our methods can work well in the situation where no hand-annotated data is provided.

## 4. Error Analysis

To show the detail of our PARE model outperforming the baseline model, we do some error analysis. We consider five error types:

- Containing: the gold entity boundary contains the predicted entity boundary.
- Be-contained: the gold entity boundary is contained by the predicted entity boundary.
- Cross: the gold entity boundary is crossed with the predicted entity boundary.
- Type-error: the gold entity boundary is the same as the predicted entity boundary, and the gold entity has a different type compared with the predicted entity.
- No-cross: there is no boundary crossing between the gold entity and the predicted entity; that is, the model predicts the unlabeled entity or forgets to predict the gold entity.

Some cases in EC are shown in Figure 3, and the rate of the LSTM-CRF model in different error types is shown in Figure 4. The main error comes from no-cross error, accounting for 40%. It may be a good choice for a model to focus on no-cross error. In Figure 5, we show the performance of the PARE model in different error types. The model incorporated distantly supervised data, and cross-domain data can greatly reduce the number of no-cross errors.

## 5. Related Work

Recently, most NER systems are based on supervised methods, such as conditional random field model and neural network model. Conditional random field model relies heavily on hand-crafted features [5, 28]. The features of the sequence can be extracted automatically in the neural network model [6, 7, 25, 29–31]. Recently, the methods of using pretraining language models have become the mainstream for solving named entity recognition. The pretraining language models [15, 32–34] can better capture the context information of the current token. In this paper, we build our models based on the LSTM-CRF model [7] and BERT [15], which are prevalent neural network models.

In the named entity recognition task, the distantly supervised data is a widely used external data [8]. A lot of methods focus on reducing the noise in the distantly supervised NER data [8, 9, 19, 35]. Yang et al. introduced a partial learning method to process the distantly supervised data [8]. Recently, Peng et al. have explored a positive-unlabeled method to process distantly supervised NER data in English [9]. Jie et al. proposed a cross-training model that can process the incomplete annotation situation [19]. A structural causal model is introduced to solve the dictionary biased problem in [35]. Zhang et al. proposed self-collaborative denoising learning methods, which jointly train two teacher-student networks in a mutually beneficial manner to iteratively perform noisy label refinery [26]. However, all these methods do not consider the NER label features. In this paper, we build our model based on [8] and propose a new label strategy using the NER label feature.

Parameters sharing method is a widely used method in cross-domain learning methods [10, 12, 27, 36]. Directly transferring cross-domain data information may lead to performance decline [37, 38]. Data selection can be useful in cross-domain learning methods for preventing negative transfer from irrelevant sentences [39, 40]. Besides, Jia and Zhang proposed the Multicell Compositional LSTM for domain adaptation. Motivated by [13], we introduce the cross-domain data selection to NER and use distantly supervised data as another external data.

In recent years, the reinforcement learning method has been used widely in natural language processing [8, 13, 41]. Feng et al. used instance selection as a reinforcement learning process in relation classification [41]. Yang et al. used the reinforcement learning method to select sentences from the distantly supervised data in NER [8]. Liu et al. used the reinforcement learning method for domain adaptation in POS tagging, dependency parsing, and sentiment analysis [13]. In this paper, we explore a PARE model that used distantly supervised data and cross-domain data simultaneously by the reinforcement learning method.

## 6. Conclusion

In this paper, we propose a PARE model that can simultaneously use distantly supervised data and cross-domain data as external data in NER. In the PARE model, first, we introduce a new label strategy to traditional partial annotated learning. The strategy can reduce the redundancy path to improve performance. Then, we introduce reinforcement learning to reduce the noise in distantly supervised data and distribution differences in cross-domain data. Finally, the model can be used in the situation where no hand-annotated data is provided. The experiments in three datasets show that our method can work perfectly.

## Figures and Tables

**Figure 1:** An example of the improved label strategy in partial learning method. The NER system tries to recognize brands and products in e-commerce data. The brown blocks are impossible tags. “B-Brand” means beginning of a brand, “I-Brand” means inside of a brand, “B-Product” means beginning of a product, “I-Product” means inside of a product, and “O” means outside of entity.

**Figure 2:** The architecture of the PARE model.

**Figure 3:** The case of different error types.

**Figure 4:** The rate of different error types in EC.

**Figure 5:** The performance of the PARE model in different error types.

**Algorithm 1:** Overall training procedure.

**Algorithm 2:** The training procedure in no in-domain hand-annotated data.

**Table 1:** The number of sentences in the different corpora.

	# rain	# Dev	# Test	# DS	# CD
EC	1200	400	800	2560	5999
News	3000	3328	3186	3722	8405
BC	3000	500	1000	3000	8405

**Table 2:** The results of models.

		EC			News			BC		
Model	Data	P	R	F	P	R	F	P	R	F
Word embedding based										
LSTM-CRF [7]	Hand	50.64	54.83	52.65	63.33	68.63	65.87	65.00	58.65	61.66
DS-PA-RL [8]	Hand + DS	58.93	60.69	59.80	75.94	76.10	76.02	73.94	78.95	76.36
CD-SHA [24]	Hand + CD	65.70	65.17	65.44	75.85	71.31	73.51	82.28	73.64	77.72
CD-ADV [14]	Hand + CD	64.09	63.49	63.79	71.03	**76.15**	73.50	72.79	74.43	73.60
DS-IPA-RL	Hand + DS	62.82	62.53	62.67	78.62	75.80	77.18	76.92	78.43	77.67
CD-RL	Hand + DS	66.82	66.67	66.74	83.63	74.30	78.69	82.30	75.81	78.92
PARE	Hand + DS + CD	**66.99**	**68.78**	**67.87**	**83.87**	76.12	**79.80**	**82.56**	**79.06**	**80.77**

BERT based										
BERT-CRF [15]	Hand	80.14	80.30	80.22	98.17	97.36	97.76	94.64	92.99	93.81
SoftLexicon [25]	Hand	81.15	81.53	81.34	98.18	97.53	97.85	94.94	93.34	94.13
SCDL [26]	Hand + DS	81.33	81.64	81.48	98.08	97.74	97.91	94.95	93.54	94.24
Multicell [27]	Hand + CD	81.82	81.69	81.75	98.17	97.76	97.96	94.89	93.65	94.27
PARE-BERT	Hand + DS + CD	**81.84**	**82.32**	**82.08**	**98.20**	**97.76**	**97.98**	**94.96**	**94.36**	**94.66**

**Table 3:** The performance of improved partial learning.

Model	Data	EC	News	BC
LSTM-CRF	Hand	52.65	65.87	61.66
LSTM-CRF	Hand + FA	51.21	61.21	71.31
LSTM-CRF-PA	Hand + PA	51.91	69.54	71.53
LSTM-IPA	Hand + IPA	**59.11**	**75.09**	**75.18**

**Table 4:** The performance of using cross-domain data by reinforcement learning method.

Model	Data	EC	News	BC
CD-SHA	Hand + 0% CD	52.65	65.87	61.66
CD-SHA	Hand + 25% CD	62.01	68.98	71.43
CD-SHA	Hand + 50% CD	64.47	71.44	74.07
CD-SHA	Hand + 75% CD	65.94	73.06	78.86
CD-SHA	Hand + 100% CD	65.44	73.51	78.23
CD-RL	Hand + CD RE	**67.46**	**78.69**	**78.92**

**Table 5:** Test results for PARE model in no hand-annotated data.

Model	Data	EC	News	BC
LSTM-PA	DS	21.78	6.30	10.34
LSTM-CRF	CD	51.60	50.98	36.36
SHA-IPA	DS + CD	53.54	62.93	57.54
PARE	DS RE + CD RE	**56.41**	**65.44**	**60.65**

## Data Availability

The dataset used in this work can be found at “rainarch/DSNER/tree/master/data,” “https://github.com/allanj/ner_incomplete_annotation/tree/master/data,” and “https://catalog.ldc.upenn.edu/LDC2013T19.”
